This article has been retracted.

# Long intergenic non-protein coding RNA 960 regulates cancer cell viability, migration and invasion through modulating miR-146a-5p/interleukin 1 receptor associated kinase 1 axis in pancreatic ductal adenocarcinoma

**DOI:** 10.1080/21655979.2020.1868742

**Published:** 2021-01-11

**Authors:** Yaoxing Huang, Qingqing Yan, Danchun Yu, Xiaojuan Sun, Shuman Jiang, Weidong Li, Lin Jia

**Affiliations:** Department of Gastroenterology, Guangzhou First People’s Hospital, School of Medicine, South China University of Technology, Guangzhou, China

**Keywords:** LINC00960, IRAK1, miR-146a-5p, pancreatic ductal adenocarcinoma

## Abstract

Long non-coding RNAs (lncRNAs) are considered as crucial regulatory factors in cancer biology. However, the biological function of long intergenic non-protein coding RNA 960 (LINC00960) in the tumorigenesis of pancreatic ductal adenocarcinoma (PDAC) is still unknown. The goal of this study is to investigate the role of LINC00960 in PDAC. Quantitative real‐time polymerase chain reaction (qRT-PCR) was used to examine the expression levels of LINC00960 in PDAC tissues and cell lines. After transfection, the loss-of-function models of LINC00960 or interleukin 1 receptor-associated kinase 1 (IRAK1) were established with BxPC-3 cells and Colo357 cells, and the malignant phenotypes of BxPC-3 cells and Colo357 cells were detected by CCK-8 assay, BrdU assay and Transwell assay, respectively. The interactions among LINC00960, miR-146a-5p and IRAK1 were predicted by bioinformatics analysis, and verified by luciferase reporter assay, RNA immunoprecipitation assay and RNA pull-down assay. The regulatory functions of LINC00960 and miR-146a-5p on IRAK1 were detected by Western blot. We demonstrated that the LINC00960 expression was increased in PDAC tissues and cell lines. Knocking down LINC00960 or IRAK1 could repress the viability, migration, and invasion of BxPC-3 and Colo357 cells. LINC00960 functioned as a molecular sponge for miR-146a-5p, and IRAK1 was verified as a target gene of miR-146a-5p. Additionally, LINC00960 could up-regulate IRAK1 expression via repressing miR-146a-5p, and the oncogenic properties of LINC00960 were partly reversed by miR-146a-5p. Our findings reveal that LINC00960 is a promoter of PDAC progression through regulating miR-146a-5p/IRAK1axis.

## Introduction

Pancreatic ductal adenocarcinoma (PDAC) emerges as a deadly cancer [1,2]. Because of its insidious symptom in early stage and strong aggressiveness, the early diagnosis of PDAC is difficult, and the 5-year survival rate is lower than 8% [3,4]. In this context, clarifying the molecular mechanism of PDAC and identifying novel biomarkers and targets for PDAC are crucial to improve patients’ prognosis.

Long non-coding RNAs (lncRNAs) have more than 200 nucleotides in length, and cannot encode proteins [5,6]. Previously, lncRNA is considered as ‘transcription noise’. However, recent studies support that lncRNA is vital in regulating diverse biological processes, including embryo development, cell multiplication, apoptosis, differentiation, gene imprinting, stress response, tumorigenesis, and so on [7–10]. Many lncRNAs regulate cancer progression, showing the potential to be biomarkers and therapeutic targets [11–15]. LINC00960 is a newly discovered lncRNA with high expression in PDAC [16], but the function and underlying mechanism of LINC00960 in PDAC are indeterminate.

MicroRNA (miRNA) features prominently in regulating the biological processes [17,18]. Reportedly, in PDAC, many miRNAs are pivotal tumor promoters or tumor suppressors [19–21]. A recent study reports that miR-146a-5p is lowly expressed in PDAC tissues and increases the chemosensitivity of cancer cells via regulating TRAF6/NF-kB p65 axis [22].

The aim of the current study is to investigate the role of LINC00960 in the progression of PDAC and to clarify the possible mechanisms. Herein, we validated that LINC00960 expression was elevated in PDAC tissues and cell lines. Importantly, LINC00960 facilitated the malignant biological behaviors of PDAC cells, and it mechanistically served as a competitive endogenous RNA (ceRNA) to regulate miR-146a-5p and interleukin 1 receptor-associated kinase 1 (IRAK1).

## Material and methods

### Tissue specimens

Tissue specimens available from 75 PDAC patients who underwent surgical resection in Guangzhou First People’s Hospital from Jan 2013 to Jan 2018 were immediately stored in liquid nitrogen at −196°C until RNA extraction. This work was approved by the Ethics Committee for Clinical Research of Guangzhou First People’s Hospital.

### Cell culture

Human pancreatic ductal epithelial cell line (HPDE) and 5 kinds of PDAC cell lines (PANC-1, BxPC-3, Capan-1, SW1990, and Colo357 cell) were obtained from the Cell bank of the Chinese Academy of Sciences (Shanghai, China). The cells were cultured in RPMI-1640 medium (Invitrogen, Carlsbad, CA, USA) with 10% fetal bovine serum (FBS, Gibco, Carlsbad, CA, USA) at 37°C in 5% CO_2_.

### Cell transfection

LINC00960 siRNA (si-LINC00960), IRAK1 siRNA (si-IRAK1), negative control siRNA (si-NC), LINC01094 overexpression plasmid (LINC00960), and negative control plasmid (NC) were obtained from GeneCopoeia (Guangzhou, China). MiR-146a-5p mimics and inhibitors were from GenePharma (Shanghai, China). They were accordingly transfected into PDAC cells to establish the cell models with Lipofectamine 2000 (Invitrogen, Waltham, MA, USA).

### Quantitative real‐time polymerase chain reaction analysis (qRT–PCR)

Total RNA extracted from tissues or cells by TRIzol reagent (Invitrogen, Carlsbad, CA, USA) was reversely transcribed to cDNA with Reverse Transcription Kit (Takara, Dalian, China). For miR-146a-5p, reverse transcription was performed with TaqMan MicroRNA Assay kit (Applied Biosystems, Foster City, CA, USA). Subsequently, qRT-PCR was performed with SYBR Premix Ex Taq (Takara, Shiga, Japan), with GAPDH and U6 as the endogenous controls. The primers are detailed in Table 1.

**Table 1.** Primer sequences

	Forward (5ʹ→3ʹ)	Reverse (5ʹ→3ʹ)
LINC00960	GCAGTAAACAGTCCTCAGCGAAG	CGGTGCCATGGAGTCTAGAAGAT
IRAK1	AGATATTGTCCTAAGTGTCAAGTCCTGA	GCCATTTCGAGCAGTGGG
GAPDH	GGAGCGAGATCCCTCCAAAAT	GGCTGTTGTCATACTTCTCATGG
U6	CGATTACGAGCAGCCTCTAGCTA	CCAGACAACGTACCGACTTTAG

### Cell counting kit-8 (CCK-8) assay

Cell viability was examined by the CCK-8 kit (Dojindo, Tokyo, Japan). Subsequent to transfection, 100 µL of cell suspension was loaded in each well of the 96-well plate (5 × 10^3^ cells/well). The cells were subsequently cultured for 24 h, 48 h, 72 h, and 96 h, and after 10 µL of CCK-8 solution was dripped into each well, the cells were incubated for 1 h. After that, the value of OD_450nm_ on a microplate reader (Promega Corporation, Fitchburg, WI, USA) was recorded.

### BrdU assay

Briefly, PDAC cells inoculated in a 96-well plate (2 × 10^3^ cells/well) were cultivated for 24 h and incubated with 10 μM of BrdU solution (BD Pharmingen, San Diego, CA, USA) for 12 h. Afterward, cells were fixed with 4% paraformaldehyde for 30 min and subsequently incubated with anti-BrdU antibody (Sigma-Aldrich, St. Louis, MO, USA) at ambient temperature for 1 h. Subsequently, the cells were immersed in PBS three times and stained with the DAPI staining solution (Beyotime, Shanghai, China) at room temperature for 30 min. Finally, the cells were observed under a fluorescence microscope, with the percentage of BrdU positive cells calculated.

### Tanswell assay

In the migration assay, the trypsinized PDAC cells were inoculated in the serum-free medium in the upper compartments (2 × 10^4^ cells/well) of the Transwell inserts (Corning, Cambridge, USA). The lower ones were loaded with medium containing 10% FBS (600 μL/well). Following 24 h of culture at 37°C, the cells on the upper surface of the membrane were wiped off with a cotton swab while the cells on the lower were fixed with paraformaldehyde for 10 min and stained for 30 min with 0.1% crystal violet solution. After the membranes were immersed in PBS and gently washed, the cells were counted under a microscope. As to the invasion assay, before the cells were inoculated, Matrigel (50 μL/well) (BD Biosciences, San Jose, CA, USA) was used to cover the membrane, and the other procedures were the same as those of the migration assay.

### Luciferase reporter assay

Wild type (WT) or mutant type (MUT) LINC00960 sequences and IRAK1 3ʹUTR sequences containing miR-146a-5p binding sites, which were amplified by PCR, were cloned into the luciferase reporter vector (Promega, Madison, WI, USA), respectively. MiR-146a-5p mimics and miR-NC were respectively transfected into HEK293 cells with LINC00960 WT or LINC00960 MUT reporter. 24 h later, the firefly luciferase activity was detected, with renilla luciferase activity as the endogenous control. Similarly, the targeting relations between miR-146a-5p and IRAK1 3ʹUTR were investigated.

### RNA pull-down assay

MiRNAs were marked by biotin through a Pierce RNA 3′ End Desthiobiotinylation Kit (Thermo Fisher Scientific, Waltham, MA, USA). Bio-miR-146a-5p and Bio-miR-NC were transfected into PDAC cells. Then, the cells were subsequently lysed and incubated with magnetic beads (Invitrogen, Carlsbad, CA, USA) before LINC00960 expression in the pulled-down complex was quantified by qRT-PCR.

### RNA immunoprecipitation (RIP) assay

RIP assay was conducted with EZ-Magna RIP Kit (EMD Millipore, Billerica, MA, USA). In short, PDAC cells were lysed in RIP lysis buffer containing cocktail (Roche Diagnostics, Shanghai, China). The supernatants were then incubated with the antibody anti-Ago2 or IgG (Millipore, Billerica, MA, USA) coupled with protein A/G magnetic beads. Then the immunoprecipitate was incubated with proteinase K. Ultimately, the RNA was extracted from the immunoprecipitate and miR-146a-5p expression was probed by qRT-PCR.

### Western blot

Cells were washed with PBS three times, and total protein was immediately extracted with RIPA lysis buffer (Biossci, Wuhan, China) on the ice. After the loading buffer was added, the protein samples were heated in boiling water for 10 min. Next, 20 µg of samples in each group was separated with sodium dodecyl sulfate-polyacrylamide gel electrophoresis and then transferred onto polyvinylidene fluoride membrane (Millipore, Burlington, MA, USA). After that, the membrane was blocked with skim milk, and incubated with the primary and secondary antibodies, and the protein bands were subsequently visualized with the enhanced chemiluminescence detection kit (Tanon, Shanghai, China). The antibodies included: anti-IRAK1 (Abcam, ab180747, 1:1000), anti-GAPDH (Abcam, ab8245, 1:3000), and secondary antibody (Proteintech, Wuhan, China, 1: 5000).

### Statistical analysis

SPSS 13.0 (SPSS, Inc., Chicago, IL, USA) was adopted for statistical analysis. All tests were performed in triplicate, and all data were in the form of mean ± standard error of mean. Data in different groups were compared with student’s *t*-test. Statistically, *P < *0.05 was meaningful.

## Results

### LINC00960 expression is up-regulated while miR-146a-5p expression is declined in PDAC tissues and cell lines

First of all, the expression characteristics of LINC00960 in PDAC was explored. qRT-PCR was employed to probe LINC00960 and miR-146a-5p expressions in 75 pairs of PDAC tissues and adjacent tissues. As against in normal pancreatic tissues, LINC00960 expression in PDAC tissues was significantly elevated (Figure 1a) while miR-146a-5p expression was down-regulated (Figure 1b). Compared with in HPDE cells, consistently, LINC00960 expression was increased in PDAC cell lines while miR-146a-5p was under-expressed (Figure 1c-d).

**Figure 1.** LINC00960 is highly expressed in PDAC samples and PDAC cell lines while miR-146a-5p was lowly expressed

A. LINC00960 expression in paired PDAC tissues and adjacent non-tumor tissues was detected by qRT-PCR (n = 75).B. MiR-146a-5p expression in paired PDAC tissues and adjacent non-tumor tissues was detected by qRT-PCR (n = 75).C. LINC00960 expression in HPDE cell line and 5 kinds of PDAC cell lines was detected by qRT-PCR.D. MiR-146a-5p expression in HPDE cell line and 5 kinds of PDAC cell lines was detected by qRT-PCR.* *P < *0.05, ** *P < *0.01, and *** *P < *0.001.

### LINC00960 knockdown represses the malignant biological behaviors of PDAC cells

Next, we conducted functional experiments to explore the effects of LINC00960 on PDAC cells. Given that LINC00960 was especially highly expressed in BxPC-3 and Colo357 cells, we selected these two cells for the subsequent experiments. We transfected two siRNAs (si-LINC00960#1 and si-LINC00960#2) and negative control (si-NC) against LINC00960 into BxPC-3 and Colo357 cells, respectively, to construct the knockdown model of LINC00960, and qRT-PCR uncovered that the efficiency of si-LINC00960#1 group was higher than that of si-LINC00960#2 (Figure 2a). Therefore, si-LINC00960#1 was used for the following assays. CCK-8 and BrdU assays were adopted to delve into the growth of PDAC cells, and Transwell assay was performed to probe the migration and invasion of PDAC cells. As shown, LINC00960 depletion markedly inhibited the malignant behaviors of both BxPC-3 and Colo357 cells (Figure 2b-f).

**Figure 2.** LINC00960 knockdown represses the proliferation, migration, and invasion of PDAC cells

A. siRNA targeting LINC00960 and negative control siRNA were transfected into BxPC-3 and Colo357 cells, respectively, and qRT-PCR was used to detect the expression of LINC00960.B. CCK-8 method was used to detect the proliferation of BxPC-3 and Colo357 cells after knocking down LINC00960.C-D. BrdU assay was used to detect the proliferation of BxPC-3 and Colo357 cells after knocking down LINC00960. Scale bar = 200 µm.E-F. Transwell assay was used to detect the migration and invasion of BxPC-3 and Colo357 cells after knocking down LINC00960. Scale bar = 200 µm.* *P < *0.05, ** *P < *0.01, and *** *P < *0.001.

### LINC00960 decoys miR-146a-5p in PDAC cells

Subsequently, the regulatory relationship between LINC00960 and miR-146a-5p was explored. Interestingly, LncBase Predicted v.2 predicted that LINC00960 contained several binding sequences for miR-146a-5p, suggesting that it could probably function as a ceRNA (Figure 3a). Notably, dual-luciferase reporter gene assay unmasked that the luciferase activity of wild-type LINC00960 reporter vector was restrained by miR-146a-5p while that of the reporter vector with three mutated binding sites was not significantly changed by miR-146a-5p (Figure 3b). Pearson’s correlation analysis elucidated that there was a negative correlation between LINC00960 and miR-146a-5p expressions in PDAC tissues (R^2^ = 0.3082, *P* < 0.001) (Figure 3c). Moreover, qRT-PCR highlighted that miR-146a-5p expression in PDAC cells was remarkably raised after LINC00960 depletion (Figure 3d). Additionally, RIP and RNA pull-down assays proved that LINC00960 could interact with miR-146a-5p in BxPC-3 cells (Figure 3e-f). These data implied that LINC00960 sponged miR-146-5p to repress its expression.

**Figure 3.** MiR-146a-5p is the target of LINC00960 in PDAC

A. The luciferase reporter vectors LINC00960-WT, LINC00960-MUT1, LINC00960-MUT2, LINC00960-MUT3, and LINC00960-MUT1&2&3 were constructed.B. The miR-146a-5p mimics were co-transfected with LINC00960-WT, LINC00960-MUT1, LINC00960-MUT2, LINC00960-MUT3, or LINC00960-MUT1&2&3 into 293 T cells, respectively. Then the luciferase activity of the cells in each group was determined.C. Pearson’s correlation analysis showed that there was a negative correlation between LINC00960 expression and miR-146a-5p expressions in PDAC tissues.D. The expression of miR-146a-5p in BxPC-3 and Colo357 cells with LINC00960 knockdown was detected by qRT-PCR.E. RNA Pull-down assay was used to detect the binding relationship between LINC00960 and miR-146a-5p.F. RIP experiment was used to detect the binding relationship between LINC00960 and miR-146a-5p.** *P < *0.01 and *** *P < *0.001.

### MiR-146a-5p targets IRAK1 in PDAC

Next, the downstream mechanism of miR-146a-5p was investigated. TargetScan database was adopted to predict the targets of miR-146a-5p, and as shown, IRAK1 was one candidate target of miR-146a-5p, whose 3ʹUTR contained two potential binding sites for miR-146a-5p (Figure 4a). Dual-luciferase reporter assay indicated that miR-146a-5p repressed the luciferase activity of wild-type IRAK1 reporter vector, but did not markedly change that of the reporter vector containing both mutated binding sites, which proved the targeting relations between miR-146a-5p and 3ʹUTR of IRAK1 (Figure 4b). We successfully transfected the mimics and inhibitors of miR-146a-5p into BxPC-3 and Colo357 cells (Figure 4c). qRT-PCR and Western blot manifested that IRAK1 expression was declined at mRNA and protein levels in cells with miR-146a-5p overexpression, but elevated when miR-146a-5p expression was inhibited (Figure 4d-e), proving that IRAK1 was a target of miR-146a-5p and could be negatively modulated by it.

**Figure 4.** IRAK1 is the downstream target of miR-146a-5p in PDAC

A. IRAK1-WT, IRAK1-MUT1, IRAK1-MUT2, and IRAK1-MUT1&2 luciferase reporter vectors were constructed.B. MiR-146a-5p mimics were co-transfected with IRAK1-WT, IRAK1-MUT1, IRAK1-MUT2, or IRAK1-MUT1&2, respectively, into 293 T cells, and then the luciferase activity of the cells in each group was determined.C. MiR-146a-5p mimic, miR-146a-5p inhibitor, and control miRNAs were respectively transfected into BxPC-3 and Colo357 cells, and the expression of miR-146a-5p in the two cell lines was detected by qRT-PCR.D. IRAK1 expression at mRNA expression level in BxPC-3 and Colo357 cells was detected by qRT-PCR after the transfection.E. Western blot assay was used to detect the expression of IRAK1 in BxPC-3 and Colo357 cells after the transfection.* *P < *0.05, ** *P < *0.01, and *** *P < *0.001.

### IRAK1 knockdown represses the viability, migration, and invasion of PDAC cells

To elaborate on the function of IRAK1 in PDAC, we transfected IRAK1 siRNA (si-IRAK1) and control siRNA (si-NC) into BxPC-3 and Colo357 cells, and Western blot indicated that IRAK1 in PDAC cells was successfully silenced (Figure 5a). CCK-8, BrdU, and Transwell assays proved that the depletion of IRAK1 observably impeded the multiplication, migration, and invasion of BxPC-3 and Colo357 cells (Figure 5b-f). These results suggested that IRAK1 could probably exert oncogenic effects in PDAC.

**Figure 5.** IRAK1 regulates the malignant phenotypes of PDAC cells

A. siRNA targeting IRAK1 and negative control siRNA were respectively transfected into BxPC-3 and Colo357 cells, and the expression of IRAK1 in the two cell lines was detected by Western blot.B. CCK-8 method was used to detect the proliferation of BxPC-3 and Colo357 cells after knocking down IRAK1.C-D. Brdu assay was used to detect the proliferation of BxPC-3 and Colo357 cells after knocking down IRAK1. Scale bar = 200 µm.E-F. Transwell assay was used to detect migration and invasion of BxPC-3 and Colo357 cells after knocking down IRAK1. Scale bar = 200 µm.** *P < *0.01 and *** *P < *0.001.

### LINC00960 regulates the malignant phenotypes of PDAC cells via miR-146a-5p/IRAK1 axis

To fathom whether LINC00960 impacts PDAC progression by modulating miR-146a-5p/IRAK1 axis, we conducted ‘rescue’ experiments. Western blot uncovered that the protein expression of IRAK1 was increased in BxPC-3 and Colo357 cells with LINC00960 overexpression, which was partially reduced by the co-transfection of miR-146a-5p mimics (Figure 6a). Functional experiments unearthed that LINC00960 overexpression significantly facilitated the multiplication, migration, and invasion of BxPC-3 and Colo357 cells while miR-146a-5p mimics partially reversed these effects (Figure 6b-d). Collectively, we concluded that LINC00960 could accelerate the progression of PDAC via regulating miR-146a-5p/IRAK1 axis.

**Figure 6.** MiR-146a-5p partially reverses the cancer-promoting effects of LINC00960 on PDAC cells

A. BxPC-3 and Colo357 cells were divided into three groups: NC+miR-con; LINC00960+ miR-con; LINC00960+ miR-146a-5p. After the transfection, Western blot was used to detect the expression of IRAK1 in the cells.B. The proliferation of BxPC-3 and Colo357 cells was detected by CCK-8 method.C. The proliferation of BxPC-3 and Colo357 cells was detected by BrdU assay.D. The migration and invasion of BxPC-3 and Colo357 cells were detected by Transwell assay.* *P < *0.05, ** *P < *0.01, and *** *P < *0.001.

## Discussion

LncRNAs partake in many cancer-related processes, including miRNA silencing, epigenetic regulation, cell cycle regulation, DNA damage response, and so on [23,24]. Little is known concerning the biological functions of LINC00960 in human diseases. Reportedly, LINC00960 expression is up-regulated in the fibroblasts of idiopathic pulmonary fibrosis, and LINC00960 negatively regulates its proliferation [25]. A recent study reports that, through up-regulating β-catenin signal, Notch signal, and Smad2/3 signal, exosome-derived LINC00960 can promote the malignant behaviors of low-grade bladder cancer cells and induce epithelial-mesenchymal transition, thus working as a potential liquid biomarker to monitor the progression of bladder cancer [26]. This study found that LINC00960 expression was up-regulated in PDAC, which is consistent with the previous report [16]. We also proved that knocking down LINC00960 observably inhibited the malignant biological behaviors of PDAC cells, implying that LINC00960 was a cancer-promoter in the PDAC progression.

IRAK1 belongs to the IRAK kinase family and its gene consists of 14 exons, which is located on X chromosome. IRAK1 is not only a part of IL1R signaling pathway, but also a downstream effector molecule of Toll-like receptor signaling pathway [27]. Additionally, IRAK1 phosphorylation is one of the important biological events in inflammatory response, and it participates in the regulation of tumorigenesis, cancer progression and drug response [28]. Targeting IRAK1/4 cascade is proved to be a promising strategy for treating various tumors, including PDAC [29]. In recent years, many studies report that IRAK1 is dysregulated in human cancers. For example, IRAK1 is overexpressed in breast cancer, which is significantly associated with the adverse prognosis of patients [30]; in lung cancer, IRAK1 high expression is relevant to the advanced clinical stage, larger tumor size, and lymph node metastasis [31]; besides, IRAK1 expression is significantly up-regulated in hepatocellular carcinoma, which modulates the stemness and drug resistance of cancer cells through regulating AP-1/AKR1B10 signaling pathway [28,32]. Notably, IRAK1 is also overexpressed in PDAC, which contributes to activating NF-κB signaling [33]. In our work, we observed that knocking down IRAK1 repressed the multiplication, migration, and invasion of PDAC cells, confirming the cancer-promoting effects of IRAK1 in PDAC.

MiR-146a-5p is a tumor suppressor in multiple cancers [34–36]. For example, in breast cancer, miR-146a-5p targets IRAK1 to restrain the malignant phenotypes of breast cancer cells [34]. The present study confirmed that miR-146a-5p expression was declined in PDAC tissues and cell lines, and this is consistent with the previous study [22]. Additionally, it was demonstrated that IRAK1 was a target of miR-146a-5p in PDAC, and this regulatory relationship is similar with that in breat cancer cells and macrophages [34,37]. We also discovered that LINC00960 negatively modulated miR-146a-5p, which, in turn, positively regulated IRAK1 expression in PDAC cells. Besides, the up-regulation of miR-146a-5p expression could partially weaken the multiplication, migration, and invasion of PDAC cells mediated by LINC00960 overexpression. These results implied that the ceRNA network consisting of LINC00960, miR-146a-5p, and IRAK1 was a novel mechanism of PDAC progression.

## Conclusion

Collectively, this study validates that LINC00960 is highly expressed in PDAC while miR-146a-5p expression is down-regulated. Functionally and mechanistically, LINC00960 participates in regulating the malignant biological behaviors of PDAC cells by modulating miR-146a-5p/PDAC axis (Figure 7). The novel ceRNA network provides potential therapy targets and diagnostic biomarkers for PDAC.

**Figure 7.** Graphic abstract: LINC00960 regulates the proliferation, migration and invasion of PDAC cells via sponging miR-146a-5p and up-regulating IRAK1

## Supplementary Material

Supplemental Material

## Research highlights

1. LINC00960 is highly expressed in pancreatic ductal adenocarcinoma (PDAC) tissues and cell lines.
2. LINC00960 regulates the proliferation and metastatic potential of PDAC cells.
3. LINC00960 functions as a molecular sponge of miR-146a-5p in PDAC.
4. IRAK1 is a target of miR-146a-5p in PDAC, and positively regulated by LINC00960.
